The article "Platelets: No longer bystanders in liver disease" was published in 2016. Journal: Hepatology.

# Platelets: No longer bystanders in liver disease

**DOI:** 10.1002/hep.28526

**Published:** 2016-04-07

**Authors:** Abhishek Chauhan, David H. Adams, Steve P. Watson, Patricia F. Lalor

**Affiliations:** ^1^ Centre for Liver Research, and NIHR Birmingham Liver Biomedical Research UnitInstitute of Biomedical ResearchBirminghamUK; ^2^ Institute for Cardiovascular Sciences, College of Medical and Dental SciencesUniversity of BirminghamBirminghamUK

## Abstract

**Growing lines of evidence recognize that platelets play a central role in liver homeostasis and pathobiology. Platelets have important roles at every stage during the continuum of liver injury and healing. These cells contribute to the initiation of liver inflammation by promoting leukocyte recruitment through sinusoidal endothelium. They can activate effector cells, thus amplifying liver damage, and by modifying the hepatic cellular and cytokine milieu drive both hepatoprotective and hepatotoxic processes. *Conclusion:* In this review we summarize how platelets drive such pleiotropic actions and attempt to reconcile the paradox of platelets being both deleterious and beneficial to liver function; with increasingly novel methods of manipulating platelet function at our disposal, we highlight avenues for future therapeutic intervention in liver disease**. (Hepatology 2016;64:1774‐1784)

**Abbreviations**
CCL: chemokine (C‐C motif) ligand
CD: cluster of differentiation
CTL: cytotoxic T lymphocyte
CXCL: chemokine (C‐X‐C motif) ligand
HGF: hepatocyte growth factor
HSC: hepatic stellate cell
HSEC: hepatic sinusoidal endothelial cell
5HT: 5‐hydroxytryptamine
IL‐6: interleukin‐6
NAFLD: nonalcoholic fatty liver disease
PDGF: platelet‐derived growth factor
TGF‐β: transforming growth factor‐β
TNF‐α: tumor necrosis factor‐α
VEGF: vascular endothelial growth factor

Traditional paradigms of platelet function focus on the role of platelets in mediating hemostasis at points of endothelial disruption or vascular damage. The archetypal platelet role, starting from adhesion to the damaged vessel wall followed by activation and aggregation triggering the clotting cascade, has been well described; and antiplatelet therapy blocking one or multiple points of the above sequence is the cornerstone of pharmacological therapy aimed at preventing arteriothrombotic vasculo‐occlusive events. However, antiplatelet therapy is often halted or suspended in patients with chronic liver disease due to the association with a coagulopathy. The relatively common occurrence of portal venous thrombosis in patients with cirrhosis argues against such a strategy, and it is likely that the bleeding diathesis associated with chronic liver disease is overstated.^1^, ^2^ Consequently, little is known about the effects of antiplatelet therapy in liver disease.

The article "Platelets: No longer bystanders in liver disease" was published in 2016. Journal: Hepatology.

A growing body of evidence derived from rodent and *in vitro* studies highlights a role for platelets far beyond the confines of hemostasis as active players in liver inflammation (Tables 1 and 2).^3^, ^4^ Platelets enter the injured liver and interact with hepatic sinusoidal endothelium, influencing effector cell recruitment and activation.^5^ These cellular interactions can result in the release of a range of up to 300 bioactive proteins (including cytokines, chemokines, growth factors, hemostatic proteins, and bacteriocidal agents^6^) from platelet α‐granules as well as bioactive lipids such as sphingosine 1‐phosphate. By releasing these bioactive molecules platelets are able to drive diverse hepatic processes ranging from necroinflammation and fibrosis to liver repair and regeneration (Table 2).^3^ Inflammatory reactions are multistep processes that can be either acute or chronic, and their sequence can vary greatly depending on the situation and organ concerned.^7^ Platelets contribute to hepatic inflammation in a disease‐specific, stage‐specific, and site‐specific manner; and it is this variance that helps to explain the pleiotropic effects of platelets in liver disease. When studying the role of platelets in liver disease, strategies employed to block platelet activation can be highly platelet‐specific (low‐dose aspirin, clopidogrel, and platelet depletion) or can also affect other cell types (cilostizol, rho kinase inhibitors, and protease‐activated receptor blockade). The latter must be taken into account when defining a role for platelets in liver disease and may explain discrepancies in the observed platelet effect in models of liver damage (see below).

**Table 1:** Summary of Models Discussed

Type of model/injury	Species	Intervention	*In vivo* or *in vitro*	Effect of intervention on liver	Reference
Viral hepatitis	Mouse	Platelet depletion	*In vivo*	Hepatoprotective	47
Viral hepatitis	Mouse	Inhibition of platelet activation	*In vitro* and *in vivo*	Hepatoprotective	12, 13, 48, 49, 50, 51
Viral hepatitis	Mouse	Blocking platelet binding to endothelium	*In vitro* and *in vivo*	Variable can be either hepatoprotective or hepatotoxic	5, 12
Isolated HSEC coculture with platelets	Human	Blocking platelet binding to endothelium	*In vitro*	Hepatoprotective (reduced effector cell recruitment)	5
Ischemia‐reperfusion	Mouse	Blocking platelet‐Kupffer cell interaction	*In vivo*	Hepatoprotective (reduction in steatosis)	42, 45, 46
Thermal injury	Mouse	Blocking platelet binding	*In vivo*	Hepatotoxic (reduced neutrophil‐mediated repair)	30
Acute cholestasis	Mouse	Inhibition of platelet activation	*In vivo*	Hepatoprotective	58, 59, 60
Chronic cholestasis	Mouse	Platelet depletion/inhibition of platelet activation	*In vivo*	Hepatotoxic (worsens fibrosis)	62, 63

The article "Platelets: No longer bystanders in liver disease" was published in 2016. Journal: Hepatology.

**Table 2:** Summary of the Various Platelet‐Derived Mediator Effects in the Liver

Context (type/stage of liver injury)	Platelet‐derived cytokine (if any) involved	Cell(s)/structure(s) involved	Effect on cell/structure	Overall effect on liver	Reference
Resection	HGF, VEGF, insulin‐like growth factor‐1	Hepatocyte	Phosphorylation of Akt and extracellular signal‐regulated kinases 1/2	Liver regeneration	65, 68, 69, 71
Resection	Sphingosine 1‐phosphate	Liver sinusoidal endothelial cells	Liver sinusoidal endothelial cells start to produce IL‐6 and VEGF	Liver regeneration	68, 69
Resection	Direct Kupffer cell adherence	Kupffer cell	Kupffer cells produce TNF‐α and IL‐6	Liver regeneration	70, 71
Hepatectomy	Serotonin	Hepatocyte	Hepatocyte proliferation	Liver regeneration	87
Carbon tetrachloride‐induced murine fibrosis	HGF	Hepatocytes, HSCs	Hepatocyte apoptosis inhibited, HSC trans‐differentiation to myofibroblasts blocked	Fibrolysis, liver regeneration	63, 74
Hepatitis C fibrosis	PDGF‐β	HSCs	HSC trans‐differentiation to myofibroblasts	Liver fibrosis	77, 79, 80
Carbon tetrachloride‐ and thioacetamide‐induced murine fibrosis	CXCL‐4	HSCs	HSC chemotaxis, chemokine expression, and immune cell recruitment	Liver fibrosis	81
Viral hepatitis	Serotonin	Sinusoidal circulation	Delayed viral clearance, enhanced T‐cell toxicity	Liver inflammation, fibrosis, and cancer	11

Max Schultz, who first described platelets in 1865 stated, “to those who are concerned with the in‐depth study of the blood of humans, the study of these cells is enthusiastically recommended.”^8^ His statement remains as pertinent as ever, particularly in a hepatic context. We are only beginning to elucidate the complex roles these cells play in maintaining liver health and driving liver disease.

## The Interaction Between Platelets and Liver Sinusoidal Endothelium Regulates Hepatic Leukocyte Infiltration

Hepatic sinusoids are lined by unique fenestrated endothelial cells, which are exposed to only minimal shear stress^5^ and have scavenger‐like functions.^9^ The unique phenotype of sinusoidal endothelium characterized by a paucity of P‐selectin expression (both constitutive and inflammation‐induced) and low levels of von Willebrand factor^5^ helps to set the hepatic vasculature apart from the majority of other endothelial beds, thus rendering the liver a specialized environment for platelet‐endothelial interactions. The combinations of signals which govern recruitment of immune cells across the sinusoidal bed are distinct from those reported in other solid organs,^5^, ^10^ and platelets may compensate for the lack of expression of attachment factors such as selectins^10^ to assist in leukocyte recruitment during inflammation. Studies in viral models of murine hepatitis,^11^, ^12^, ^13^ human liver regeneration, and ischemia‐reperfusion injury^14^ demonstrate platelet sequestration within hepatic sinusoids. *In vitro* studies with human hepatic sinusoidal endothelial cells (HSECs) demonstrate that platelet adhesion is partly integrin (GPIIb/IIIa and αVβ3)‐mediated,^5^ with the precise location of hepatic platelet adhesion varying dependent on the type of injury. For instance in ischemia‐reperfusion injury platelets are selectively sequestered to the periportal and midzonal sinusoidal endothelium.^5^ Bound platelets activate isolated HSECs to express chemokine (C‐X‐C motif) ligand 8 (CXCL‐8) and chemokine (C‐C motif) ligand 2 (CCL‐2), thereby promoting neutrophil and lymphocyte recruitment (Fig. 1).^5^ Studies in rats have revealed that platelet‐driven leukocyte recruitment results in hepatic damage during systemic endotoxemia and that platelet‐endothelial interactions precede and drive leukocyte adherence.^15^ Furthermore, leukocytes themselves can also recruit platelets to the liver. Models of ischemia‐reperfusion injury in mice reveal the ability of cluster of differentiation 4 (CD4) T cells to activate endothelial cells, thus driving platelet recruitment to the liver sinusoids (Fig. 1). The end result is a self‐perpetuating cycle of microvascular dysfunction and hepatocellular injury.^16^ A schematic summarizing platelet HSECs and lymphocyte interactions is shown in Fig. 1.

The article "Platelets: No longer bystanders in liver disease" was published in 2016. Journal: Hepatology.

**Figure 1:** (A,B) Activated platelets bind to the endothelium, causing the endothelium to up‐regulate and secrete CXCL8 and CCL2. These chemokines recruit T cells and neutrophils to the endothelium. (C) T cells use the platelets to bind to the endothelium. Platelets use CD44 to bind sinusoidal hyaluronic acid, allowing T cells to survey the liver for viral antigen.

## Platelet Interactions With Myeloid Cells

Platelet interaction with myeloid cells, particularly macrophages and neutrophils, has been extensively investigated in the context of cardiovascular disease, thrombosis, and atherosclerosis.^17^, ^18^, ^19^ The role platelets play in innate immunity and inflammation through interaction with myeloid cells is, however, frequently overlooked.^20^ These inflammatory and immune interactions are highly relevant to liver disease because neutrophils and macrophages play central roles in liver injury, fibrogenesis, and regeneration.^21^, ^22^, ^23^, ^24^

In both humans and mice, neutrophils are recruited and activated during the acute phase of liver inflammation in response to a variety of injuries.^24^, ^25^ Cholestatic liver injury,^26^ alcoholic hepatitis,^23^, ^27^ drug‐induced injury,^28^ and chemical‐induced injury^29^ are all associated with neutrophil recruitment. The molecular and cellular mechanics of neutrophil recruitment to sites of liver injury involve specific chemokines and activation through damage‐associated molecular patterns.^30^ Platelets not only activate and recruit neutrophils to inflamed tissue^31^ but also interact with neutrophils to trap microbes in neutrophil extracellular traps,^32^ a process known to promote neutrophil‐mediated hepatotoxicity. Researchers note enhanced platelet‐neutrophil interaction within liver sinusoids during endotoxemia^33^ and have hypothesized that circulating platelet:neutrophil aggregates can perpetuate neutrophil activation, thus driving end organ damage in patients with cirrhosis.^34^

The article "Platelets: No longer bystanders in liver disease" was published in 2016. Journal: Hepatology.

Although the accepted paradigm is that, regardless of initial insult, neutrophils recruited to the site of liver damage exacerbate liver damage,^24^ recent evidence suggests that they may also have anti‐inflammatory and restorative properties. For example, platelets have recently been shown to physically “pave the way” for neutrophils to enter the liver during sterile liver injury to aid repair (Table 1).^35^

Macrophages are involved in both driving and helping resolve liver disease, being capable of mediating liver injury, fibrosis progression, fibrosis resolution,^36^, ^37^ pathogen clearance, and regulation of inflammation.^22^ Distinct macrophage subsets are activated and recruited by factors expressed in the injured liver and help shape the nature and outcome of liver injury. Platelets have an important role in regulating these processes; platelet‐derived CXCL4 and microparticles induce patterns of macrophage activation consistent with tissue repair^38^ and matrilysis,^39^ respectively. *In vitro* studies using human cells demonstrated the ability of platelet‐derived CXCL4 to induce differentiation of blood monocytes to tissue macrophages.^40^ These macrophages then switch to a proinflammatory phenotype on interacting with activated platelets at sites of tissue inflammation.^41^ In the liver, Kupffer cell‐platelet interactions are important determinants of the outcome in ischemia‐reperfusion injury. During the early period of an ischemic insult, platelets sequester in the liver, with most adhering to Kupffer cells,^42^ most likely through the interactions between platelet CLEC‐2 and macrophage podoplanin, which is up‐regulated under inflammatory conditions.^43^, ^44^ The interaction between platelets and Kupffer cells provides bidirectional signals which together drive tissue injury; reducing platelet‐Kupffer cell binding ameliorates hepatic inflammation in steatotic livers of rodents.^45^ During ischemia‐reperfusion injury platelet‐Kupffer cell interaction precedes and initiates leukocyte accumulation, sinusoidal dysfunction, and the iterative inflammation which eventually results in liver failure.^46^

The article "Platelets: No longer bystanders in liver disease" was published in 2016. Journal: Hepatology.

## Disease‐Specific Platelet Contribution

### VIRAL HEPATITIS: ARE PLATELETS A PRIMARY MEDIATOR OF VIRAL HEPATITIS?

The generation of virus‐specific T cells is an important determinant of the outcome of viral hepatitis. Lang et al. described how platelets aggravate viral hepatitis in mice through the secretion of serotonin, which results in hepatic sinusoid microcirculation failure, delayed viral clearance, and enhanced cytotoxic T lymphocyte (CTL)‐mediated liver damage.^11^ Several other murine studies also demonstrate that depleting platelets attenuates CTL‐mediated liver damage^47^; platelet reconstitution is able to restore intrahepatic T‐cell accumulation and cytotoxicity. The need for platelet activation is shown by studies in which reconstituting platelet‐depleted mice with platelets rendered resistant to activation by treatment with prostaglandin E_1_ did not restore T cell‐mediated liver damage (Table 1).^12^ Platelet activation inhibitors including aspirin and clopidogrel also reduce acute hepatic necroinflammation and intrahepatic antigen‐specific CTL accumulation during murine viral hepatitis.^48^, ^49^, ^50^ Strikingly, reducing intrahepatic CTL accumulation in mice by long‐term low‐dose aspirin therapy serves to ameliorate the consequences of chronic hepatitis including fibrosis and the development of hepatocellular cancer.^13^, ^51^

As with most physiological processes, a degree of redundancy is observed when describing the molecular basis of platelet and hepatic sinusoid interaction. There are multiple mechanisms through which platelets interact with HSECs, and blocking one route does not totally abrogate binding. Thus, although blocking integrins GPIIb/IIIa and αVβ3 reduces platelet‐sinusoidal binding *in vitro* by almost 50%,^5^ other molecules such as platelet CD44 are also important. *In vivo* murine experiments examining the mechanisms of liver immunosurveillance by T cells reveal that platelets adhere to sinusoidal hyaluronan by CD44 promoting attachment of flowing effector CD8 T cells to the vessel wall (Fig. 1).^52^

### THE PLATELETS OF NONALCOHOLIC FATTY LIVER DISEASE

The hepatic manifestation of the “metabolic syndrome” is nonalcoholic fatty liver disease (NAFLD).^53^ Platelets already have well‐described roles in the vascular complications of the metabolic syndrome and atherosclerosis; a role for platelets in NAFLD is also beginning to emerge. Mean platelet volume, a surrogate marker of platelet turnover, is consistently higher in patients with NAFLD^54^; and there is a direct correlation between mean platelet volume and histological severity of hepatic inflammation and fibrosis.^55^ *In vivo* murine studies support a role for platelets in fatty liver disease.^56^ These studies, however, need to be interpreted with caution as the antiplatelet drug cilostizol, demonstrated to have the most marked effect on reducing hepatic steatosis, inflammation, and fibrosis in mice on high‐fat/high‐calorie or choline‐deficient diets,^56^ has numerous “nonplatelet” effects. Data regarding antiplatelet therapy and liver disease in humans are generally lacking, but a large recent cross‐sectional analysis suggests that regular aspirin use may be associated with a lower prevalence of NAFLD.^57^

The article "Platelets: No longer bystanders in liver disease" was published in 2016. Journal: Hepatology.

### DUAL ROLES FOR PLATELETS IN CHOLESTATIC LIVER INJURY

Depletion of platelets protects against cholestasis‐induced hepatic inflammation and injury, suggesting that platelet interactions within the microvasculature may be important in cholestasis‐induced liver damage.^58^ A variety of strategies designed to block platelet function have similar effects in acute murine cholestatic injury. Rho‐kinase inhibitors reduce liver damage in bile duct ligation models of cholestasis,^59^ while platelet depletion reduces hepatic necroinflammation in response to alpha‐naphthylisothiocyanate‐mediated cholestatic liver injury. The alpha‐naphthylisothiocyanate cholestatic model further highlights the importance of platelet‐mediated neutrophil recruitment in driving liver damage because platelet inhibition also markedly reduces intrahepatic neutrophil accumulation and hepatic inflammation.^60^

However, as with other injury models, the role of platelets in cholestatic liver injury evolves with the development of chronicity. Although perpetuating acute inflammation early on, in the late stages of cholestasis platelet activation is hepatoprotective. Inducing a thrombocytopenia in mice during the latter stages of chronic cholestasis therefore worsens liver function by causing hepatic fibrosis (Table 1).^61^ Studies in protease‐activated receptor 4‐deficient mice suggest that it is probably platelet activation resulting in platelet matrix metalloproteinase secretion and fibrolysis that underlies their observed hepatoprotective effect in chronic cholestasis (Table 1).^62^, ^63^

## Liver Regeneration and Fibrosis: Two Sides of the Same Platelet?

### PLATELETS DRIVE LIVER REGENERATION AND INHIBIT FIBROSIS

Platelets are critical regulators of liver regeneration. After hepatic resection, platelets sequester at the resection margins and orchestrate the complex ontogenic processes necessary for functional hepatic architecture to develop.^64^ The first suggestion that platelets may have a role in liver regeneration came from studies in rats, where thrombocytosis was observed to aid liver regeneration through hepatocyte growth factor (HGF).^65^ Subsequently, it was shown that platelets are potent mediators of liver regeneration; thrombopoietin‐induced thrombocytosis experiments have demonstrated improved survival in rodent models of partial hepatectomy ordinarily lethal (e.g., 90% hepatectomy)^64^ or situations where regeneration has been traditionally thought of as undermined such as cirrhosis.^66^ Additionally, thrombocytopenia inhibits liver regeneration in partially hepatectomized mice.^14^

The article "Platelets: No longer bystanders in liver disease" was published in 2016. Journal: Hepatology.

Platelet‐mediated hepatic regeneration is dependent on their ability to bind to sinusoidal endothelium, interact with Kupffer cells, and traverse the space of Disse to interact with the hepatocytes,^67^ as described below and shown schematically in Fig. 2.

**Figure 2:** (A) Regeneration. Platelets stimulate liver regeneration by three simultaneous interactions. (1) Kupffer cells: On binding platelets, Kupffer cells become activated and produce TNF‐α and IL‐6. (2) Hepatocytes: Platelets directly stimulate hepatocyte growth and proliferation through HGF, insulin‐like growth factor‐1, and VEGF. (3) Sinusoidal endothelial cells: Activated platelets produce sphingosine 1‐phosphate, which promotes liver regeneration through phosphorylation of Akt and extracellular signal‐regulated kinases 1/2. (B) Fibrosis. Platelets produce TGF‐β, PDGF‐β, and CXCL4 to aid conversion of hepatic stellate cells into collagen‐producing myofibroblasts. Abbreviations: ERK, extracellular signal‐regulated kinase; IGF‐1, insulin‐like growth factor 1; S‐1‐P, sphingosine 1‐phosphate.

*In vitro* studies with cultured HSECs reveal that platelets promote endothelial production of interleukin‐6 (IL‐6) and vascular endothelial growth factor (VEGF) through sphingosine 1‐phosphate. These two proteins simultaneously inhibit apoptosis and stimulate hepatocyte proliferation (Fig. 2),^68^, ^69^ thus providing important cues in the regenerating liver.

Kupffer cells closely interact with platelets within the hepatic sinusoids in the period after hepatectomy, resulting in bidirectional activation.^67^ This has two consequences during hepatic regeneration. Firstly, Kupffer cells begin producing tumor necrosis factor‐α (TNF‐α) and IL‐6, cytokines critical to liver regeneration.^70^, ^71^ Secondly, activated platelets begin to move through the sinusoidal endothelium, entering the space of Disse (most likely attached to Kupffer cells) to directly exert a promitogenic influence on hepatocytes.^72^ Platelets release HGF, VEGF, and insulin‐like growth factor‐1, which stimulate pro‐proliferative pathways critical to hepatocyte survival and differentiation through phosphorylation of Akt and extracellular signal‐regulated kinases 1/2 (Table 1 and Fig. 2).^71^

The article "Platelets: No longer bystanders in liver disease" was published in 2016. Journal: Hepatology.

The prohepatic or regenerative effects of platelets extend to inhibiting fibrosis. Thus, in parallel with their mitogenic effect on hepatocytes, platelets suppress fibrogenesis and initiate fibrolytic pathways. The role of platelets in reducing cholestasis‐associated fibrosis in mice has been discussed above.^61^, ^73^ Human platelets inhibit liver fibrosis in severe combined immunodeficiency mice by secreting HGF, which exerts antifibrotic effects by simultaneously blocking hepatic stellate cell (HSC) activation and promoting matrix metalloproteinase 9 expression (an enzyme known to drive fibrolysis).^63^, ^74^

### BUT PLATELETS CAN ALSO DRIVE FIBROSIS

Liver repair and regeneration require both pro‐proliferative and antiproliferative signals to coordinate tissue repair. Platelets play a dual role: in addition to their ability to suppress fibrogenesis and drive hepatic mitogenesis, under certain conditions platelets have the potential to diminish hepatocyte regeneration and exacerbate fibrosis.^39^, ^75^

Rodent studies reveal that platelet lysates have the ability to drive profibrotic cytokine secretion by HSCs *in vitro*.^76^ Human studies substantiate this finding as human platelets contain the potently fibrogenic transforming growth factor‐β (TGF‐β) and platelet‐derived growth factor‐β (PDGF‐β)^4^, ^77^, ^78^ (Fig. 2), both of which induce HSC trans‐differentiation *in vitro* to fibrogenic myofibroblast‐like cells.^4^, ^77^, ^79^ Furthermore, activated HSCs up‐regulate the PDGF‐β receptor and are found in close apposition with sequestered sinusoidal platelets in patients with hepatitis C cirrhosis.^80^

Another platelet‐derived cytokine implicated in liver fibrosis is CXCL4. Hepatic CXCL4 levels increase proportionately to fibrotic burden, and CXCL4^‐/‐^ mice display markedly less hepatic fibrosis in response to injurious stimuli than their wild‐type counterparts.^81^ Similar findings have been reported in human chronic liver disease; patients with advanced fibrosis have high intrahepatic and serum concentrations of CXCL4.^81^ A schematic summarizing the platelet role in liver regeneration and fibrosis is shown in Fig. 2.

Little is known about the effects of portal hypertension‐induced thrombocytopenia in chronic human liver disease. In keeping with murine studies,^61^ however, the resolution of platelet count in splenectomized patients improves liver function in cirrhosis.^82^

The article "Platelets: No longer bystanders in liver disease" was published in 2016. Journal: Hepatology.

### PLATELET‐DERIVED SEROTONIN: A POISONED CHALICE?

Platelet‐derived serotonin further exemplifies the complexity and diverse roles of platelets in liver pathophysiology.

Most of the total‐body serotonin is found in the gut, specifically within the enterochromaffin cells and enteric neurons.^83^ Platelets tightly regulate the small amount of free serotonin in the blood, using the serotonin reuptake transporter.^84^ Consequently, they contain about 95% of the total plasma serotonin and have high intracellular serotonin concentrations.

Platelets mediate vasoconstriction within the hepatic sinusoidal microcirculation using serotonin to mediate HSECs or HSC contraction,^85^ resulting in hepatic hypoperfusion.^86^ The vasoactive effects of platelet‐derived serotonin are likely to be the main contributors to the effect seen by Lang et al.^11^ in viral hepatitis because Guidotti et al. report that serotonin is not required for virus‐specific T‐cell accumulation in the liver.^52^

In contrast to its nonspecific role in perpetuating viral hepatitis, serotonin has a central and relatively well‐defined role in liver regeneration. Platelet‐derived serotonin interacts with both hepatocytes and HSCs, and it is the ability of serotonin to modulate the phenotypic plasticity of these cells that helps explain the effects of serotonin in liver regeneration after injury.

In the early phase of murine liver injury, immediately after partial hepatectomy, an up‐regulation of 5‐hydroxytryptamine (5HT) 2A and 2B messenger RNA is observed in the liver. Antagonism of these serotonin receptors (5HT 2A and 2B) inhibits liver regeneration.^87^ Furthermore, serotonin receptor (5HT 2A, 2B, and 2C subtypes) antagonism using ketanserin completely suppresses liver regeneration after partial hepatectomy^88^ in mice, and mice deficient in tryptophan hydroxylase (the enzyme necessary for serotonin production) exhibit impaired liver regeneration.^14^ Further proregenerative effects of platelet‐derived serotonin are seen in its ability to rescue small for size livers following transplantation^87^, ^89^ and reversing age‐related liver pseudocapillarization.^90^

In the late stages of liver injury, however, HSCs participate in termination of the regeneration process and actually promote fibrosis. At this time point, platelet‐derived serotonin interacts with HSC 5‐HT 2b receptors stimulating HSC TGF‐β expression.^77^, ^91^ Furthermore, activated HSCs assume a fibrogenic phenotype and up‐regulate three subtypes of serotonin receptor (5‐HT 1B, 2A, and 2B), antagonism of which results in HSC apoptosis aiding fibrosis resolution.^92^

The article "Platelets: No longer bystanders in liver disease" was published in 2016. Journal: Hepatology.

Overall the contribution of platelets in general and platelet‐derived serotonin specifically favors regeneration or liver repair, but it is important to note that regeneration and fibrosis are both part of the repair response to injury. The ability of platelets to influence both processes demonstrates how pleiotropic these cells are. Platelets are crucial for regeneration to occur, and after acute liver injury, this is their dominant contribution. However, as liver damage approaches chronicity, platelets participate in fibrogenesis and actively block regeneration, in part through serotonin‐driven TGF‐β expression. Whether platelets provide predominantly promitogenic or profibrotic signals is determined by the cellular and cytokine microenvironment specific to the stage and type of liver injury.

## Conclusion and Future Directions

Platelets play a central role both in liver homeostasis and in the response of the liver to injury. The complexity of this role is becoming increasingly apparent as advances in genomic, proteomic, and transcriptomic analyses enable researchers to define roles for platelets beyond hemostasis (Table 1).

Recent work suggests that aspirin reduces the risk of liver fibrosis in patients who have been transplanted for hepatitis C.^93^ Mechanistically, aspirin and clopidogrel inhibit dense granule release, blocking serotonin among other small molecules. These drugs also inhibit the expression of α‐granule‐stored proteins that are involved in heterotypic interactions between platelets/leukocytes and the endothelium including P‐selectin and CD40L.^51^ Reducing platelet activation alters how immune‐mediated chronic hepatitis progresses, impacting even cancer development.^51^ Modulating the way platelets deliver serotonin to the liver sinusoid during injury may also be open to therapeutic manipulation. Given its propensity to aggravate viral hepatitis,^11^ one would assume blocking serotonin would beneficial in chronic hepatitis. However, when studied in the context of nonviral hepatic inflammation, for example, acute liver injury due to acetaminophen toxicity, serotonin deficiency worsens outcome,^94^ possibly through the ability of serotonin receptor 5HT 2A to reduce TNF‐α‐mediated inflammation.^95^ Serotonergic agonists may therefore be of therapeutic benefit during acute nonviral liver inflammation, but little is known about the effect of drugs such as selective serotonin reuptake inhibitors on liver inflammation or regeneration.

Given the complex and dualistic roles played by platelets outlined above, the evidence for recommending when to use antiplatelet therapy in liver disease is far from complete. It is important that future preclinical studies delineate the precise molecular basis of platelet activation and the functional consequences in the context of liver injury. Only by understanding the disease and disease stage‐specific platelet contribution will we be able to design logical and safe interventions with antiplatelet therapies. Evolving understanding of how platelets mediate inflammatory damage, modulate vascular integrity, and interact with leukocytes^96^, ^97^ suggests there may well be a role for antiplatelet therapy in treating inflammatory and fibrotic liver disease.

The article "Platelets: No longer bystanders in liver disease" was published in 2016. Journal: Hepatology.

With the repertoire of antiplatelet therapy already available, multiple potential avenues of novel treatment are possible. As Friedman et al. aptly state, “Still, it is heartening that platelets, which have always been present in the scene of hepatic injury during disease, are now also considered as actors in the scene.”

Author names in bold denote shared co‐first authorship.
